This article has been retracted.

# The impact of trade and financial expansion on volatility of real exchange rate

**DOI:** 10.1371/journal.pone.0262230

**Published:** 2022-01-21

**Authors:** Zhe Chen

**Affiliations:** School of Economics, Zhejiang University, Hangzhou, China; Ministry of Natural Resources North Sea Bureau, CHINA

## Abstract

With the steady progress of China’s opening-up policy, how to avoid the financial risks brought by opening-up is a valuable research topic at present while promoting economic development. As an innovative business model connecting the real economy and the virtual economy, the Internet of Things (IoT) finance provides standardized technical support for the expansion of trade and finance. In financial data analysis, deep learning (DL) has become an important means to predict financial market movements, process text information and improve trading strategies. Analysis is conducted on the influence of trade and financial opening on the volatility of real exchange rate. Through the empirical test of panel data of 45 major countries in the world, the pooled ordinary least square (OLS) method and instrumental variable method are used to evaluate the influence of trade and financial opening of sample countries on the volatility of real exchange rate. The main conclusions are that trade openness is negatively correlated with the volatility of real exchange rate, and financial openness is positively correlated with the volatility of real exchange rate. A certain reference is provided for reducing the fluctuation of real exchange rate in the process of opening to the world.

## 1. Introduction

The financial liberalization is a theory of economic development put forward by western economists in the 1970s, which gives birth to developing countries’ financial reform titled as “financial liberalization” [1]. In the process of economic development of developing countries, the main reasons for the slow economic development are insufficient capital resources and distorted financial markets. Only when the government deregulates the financial market can currency and relative price play a role [2]. The reform of financial system is theoretically promoted by financial liberalization, as well as that the government should lose its restrictions on financial institutions and markets, the financing function should be improved to avoid depending on foreign investment, and the interest rate and exchange rate should be deregulated to meet the actual need of the domestic market. In this way, the relationship between supply and demand of foreign exchange can be reflected in the exchange rate. The domestic savings rate should be increased to eventually realize the curb inflation and economic growing [3]. Financial liberalization promotes the economic and financial growth. However, financial liberalization intensifies the vulnerability of finance system, and the recession crisis caused by financial vulnerability in turn.

Artificial intelligence (AI) has been used in every kind of scenes due to the development of technologies such as Big Data (BD) and parallel computing, which plays a significant role in the industry to realize profound economical changes and development of society. DL is frequently used in the financial reform, which is the key technology to process diversified AI tasks and the core instrument to break the bottleneck of AI development. DL can realize accurate volatility forecasting and it is also frequently adopted in the price forecasting of all kinds of financial assets, such as stocks, futures, and bonds. Better design and other optimization should be conducted on the disparate DL structures for better forecasting results. Comparison of the prediction effect has been made many scholars in the application of DL with that of other traditional models. The conclusion is that prediction accuracy can be improved by the DL method. The traditional extensive operation mode has been difficult to adapt to the production relations in the era of science and technology finance. As a new core productivity, IoT technology may create an innovative business model and open the second curve of trade financing. In the era of "Internet of Everything", supply chain financial services will achieve a fundamental change from online to presence, and business side (B-side) financial services will be able to be carried out in real time in the scene.

With changes constantly happening to the world economy, economic globalization has become the basic feature of the current era. While all countries are developing in this environment, they also share the risk. Under the environment of economic opening, each country mainly exchanges through international trade and capital flow, which also makes the level of bilateral trade and multilateral trade open continuously improve [4,5]. At the same time, due to the integration of international finance and capital market caused by economic opening, the degree of trade and financial opening of each country is significantly improved. Data show that between 1980 and 2015, the output of each country increased by 2.7 times, while the total amount of global trade increased by 4.3 times. The growth of trade far exceeds the growth of output, which is an important performance of trade opening [6]. Nilavongse et al. (2020) investigated the impact of international economic policy uncertainty shocks on the UK’s economy, and confirmed that interference with domestic economic uncertainty was an important factor the volatility of real exchange rate [7]. Sheikh et al. (2020) used a nonlinear autoregressive distributed lag model to analyze the relationship between macroeconomic fluctuations and stock indexes before and after the 2008 economic crisis, and finally determined that the relationship between macroeconomic fluctuations and stock prices is essentially asymmetric [8]. Although the above research has achieved some valuable results, it has not yet solved the endogenous problem between opening up and the volatility of real exchange rate. Therefore, an in-depth analysis is conducted on this research gap.

For China, the implementation of reform and opening up is the beginning of trade and financial opening up, and gradually develop and improve. But in the process of opening up, the volatility of exchange rate is also affected, and great changes have taken place. In the 1970s, after the Bretton Woods system broke down, the whole world experienced frequent the exchange rate volatility, and the international financial market became increasingly volatile. The international monetary system is an important defense line to effectively prevent financial market risks. At the beginning of a financial crisis, abnormal volatilities in the foreign exchange market usually occur, leading to a currency crisis, which then develops into currency and securities market oscillations, eventually affecting the normal operation of the Real Economy. Therefore, in the early stage of the formation of systemic financial crisis, the abnormal volatility of exchange rate can be used as a starting signal, and maintaining the stability of exchange rate plays an important role in preventing financial crisis. The theoretical model is combined with the empirical analysis to deeply study the measures to ensure the exchange rate stability in the process of trade and financial expansion and opening up, to provide reference for preventing financial risks caused by external shocks and formulating economic policies. The innovation is to solve the endogenous problem between trade openness, financial openness, and the volatility of real exchange rate by instrumental variable method.

## 2. Analyses on the influence of trade and financial opening on the volatility of real exchange rate

### 2.1 Related factors of real exchange rate volatility

The exchange rate of a country is published by the country’s monetary authority, which is also called nominal exchange rate. The nominal exchange rate of foreign exchange bank can be expressed by the direct pricing method or the indirect pricing method [9]. Real exchange rate is determined according to the adjusted nominal exchange rate, which is used to calculate the relative price level between two different countries. The level of a country’s goods and services in the international market can be reflected in the real exchange rate more precisely than the nominal exchange rate. Therefore, the research on the exchange rate mainly focuses on the real exchange rate [10]. The volatilities of a country’s foreign exchange rate directly affect its import and export trade, economic structure, and production layout. Generally, the decrease of the ratio of local currency to foreign currency, can function as accelerating exports and restraining imports. If local exchange rate declines, it is beneficial to imports and unfavorable to exports.

According to The Law of One Price, the value of diverse commodities accords the same among countries. In a free market, where two parties of the trade do not need to pay for transport of the commodity and there are not official trade barriers, no matter where the same commodity is sold to and priced under the same currency, its price should be equal [11]. According to the traditional theory, the main reason for the volatility of real exchange rate is the deviation between tradable goods and The Law of One Price. Specifically, the basic factors that cast influence on the volatilities of exchange rate mainly include the following several aspects.

First, balance of payments and foreign exchange reserves: balance of payments can directly affect the change of a country’s exchange rate. A country will see the foreign exchange rate of its currency rising, if there is a balance of payments surplus, otherwise, the country will see the exchange rate declining. Capital will flow in, if the quantity of export is larger than that of the import in the balance of payments. And when capital flow in, the country’s currency will become more required by the international market. However, if the quantity of the import is greater than that of the export of the country, capital will flow out, which means the international market needs less currency of the country, and the local currency in the country will depreciate.

Second, interest rate: as the basic index to reflect the lending situation of a country, interest rate almost decides the volatility of exchange rate. The level of interest rate is intimately connected with the international capital flow. Capital flows in the countries with high interest rate, and flows out the countries with low interest rate. Capital flow will alternate the supply-demand relationship in the foreign exchange market, thus affecting the volatility of foreign exchange rate. In general, a country’s interest rate rises then its currency becomes popular.

Third, inflation: inflation will cause the decline of the currency exchange rate in a country. And the exchange rate will not increase until the inflation is eased. Inflation damages the purchasing power of the currency in a country and weakens the competitiveness of the currency in commodities export. While the commodities import increases simultaneously, and a psychologically negative impact of the currency is casted on the foreign exchange market thus weakening the credit status of the currency [12].

Fourth, political situation: a country’s political changes or an international event may influence the foreign exchange market. The political changes refer to significant events such as political conflicts, military conflicts, elections, and regime changes. Exchange rate is fragile to these political factors, but it will get back to the normal status soon after being influenced by politics.

Fifth, economic growth rate: Gross Domestic Product (GDP) reflects the overall national income and expenditure of a country. Some parts of the requirements of people for imported commodities come from the increase of the standard of income. However, the domestic currency will therefore devaluate [13]. The phenomenon that a country’s people put more money into investment and consumption is referred to the growth of expenditure. It helps promote a country’s production industry and competitiveness of products in the international market, and stimulate a country’s commodities exports.

### 2.2 The theory of the influence of trade and financial opening on the volatility of real exchange rate

Trade opening refers to strengthening a country’s foreign trade, including opening trade barriers, reducing tariffs and other measures. The degree of trade opening is generally measured by the degree of dependence on foreign trade, which is expressed as the proportion of total import and export trade in GDP (Gross Domestic Product) in a year, and is an important indicator to evaluate the degree of market trade opening of a country. Financial opening refers to the process of gradual opening of a country’s financial system to the outside world, including the opening of capital and financial accounts and the opening of financial services [14]. The degree of financial opening can be measured by the proportion of a country’s external assets to GDP. The trend of trade opening and financial opening of major countries in the world from 1980 to 2015 are shown in Figs 1 and 2, respectively. In recent years, the strength of global trade opening has gradually increased, which shows that economic activities of more countries have been facing the global market.

**Fig 1:** Trade opening trend.

**Fig 2:** Financial opening trend.

The sharp volatility of exchange rate will lead to the turbulence of foreign exchange and stock market, and then affect the macro economy, which will have a profound impact on the real economy. Therefore, the sharp volatility of exchange rate is not conducive to economic growth and international trade. At this stage, the core contents of promoting financial opening in China mainly include financial industry opening, exchange rate marketization reform, RMB capital account free exchange, and RMB internationalization [15–17]. With regard to the impact of trade opening on the volatility of real exchange rate, it is generally believed that after trade opening, the price of imported goods will be reduced, the trade barriers between countries will be reduced, and the volatility of real exchange rate will be reduced. Financial opening mainly includes three parts: financial industry opening, exchange rate marketization, and capital account liberalization. Financial liberalization is considered to be the cause of higher exchange rate uncertainty, and the level of financial opening determines the long-term stability of the real exchange rate. The more diversified the economic structure of a country is, the lower the debt equity ratio is, and the more stable the real exchange rate volatility of the country is [18].

### 2.3 Intelligent trade and financial market supported by “deep learning + Internet of Things”

In the financial field, intelligence is an important direction of the development of the financial industry. Intelligent investment, intelligent research and intelligent investment will be the manifestations of intelligent finance, and the key to realize these concepts is how to realize ’intelligence’. The successful application of DL in other fields provides a good reference for the development of intelligent finance. From the perspective of type, financial data are mainly time series data. Time series data often has three characteristics: First, it usually has a lot of noise and high dimension characteristics; second, it is uncertain whether the obtained information is sufficient to predict the future trend; the third feature is the most direct manifestation of the time-varying data. The advantage of DL in the financial field is that as long as the data related to prediction problems can be included in the model, not limited by the data dimension. Moreover, considering the nonlinear and complex interaction between input data, compared with the traditional model, the intra-sample fitting can be improved, and the over-fitting problem can be effectively avoided.

The credit relationship in traditional trade financing is dominated by subjective credit. Bank provides financing support to enterprises by investigating the operation status of enterprises and conducting credit rating. Its decision-making depends more on subjective judgment and experience accumulation. The defect of subjective credit model lies in the incomplete control of enterprise information. The working principle of the data created by the Internet of Things is similar to that of financial technology data in recent years. The data types of both industries have simple messages: a timestamp, an identifier, and net load information. Therefore, for financial technology practitioners, the nature of the size and type of transmission information of the Internet of Things data packets is very similar to that of financial technology. If the IoT equipment and technology are directly linked to the whole process of purchasing, production, processing and sales of the production scene of the borrowing enterprise, the information distortion and subjective factors can be eliminated by real-time and objective scene data information for pre-loan investigation, loan approval and post-loan management. These multi-dimensional objective information sources can truly reflect the operating strength and operating status of borrowing enterprises, which has important reference value for dynamic risk identification of banks and lays a data foundation for banks to establish an objective credit system.

## 3. Empirical test

### 3.1 Research data and methods

In order to empirically test the impact of trade and financial expansion on volatility of real exchange rate, the panel data of 45 major countries in the world from 1981 to 2015 were taken as the research sample to conduct benchmark empirical test. Data comes from the World Bank and World Development Indicators database. Among them, 21 were developing countries and 24 were developed countries. After data processing, the final data set used includes 313 observations.

The variables were divided into explanatory variables (trade opening and financial opening), explanatory variables (real exchange rate volatilities), and control variables (factors affecting real exchange rate volatilities). Among them, for the measurement of explanatory variables, policy indicators and outcome indicators were considered, respectively. Through the policy indicators of trade opening, the degree of trade opening of a country can be judged, and through the outcome indicators of trade opening, the impact of trade types on the real exchange rate volatilities can be examined, expressed as the percentage of total import and export in GDP. The financial opening policy index is also the Chinn-Ito capital opening index, which is calculated according to different types of restrictions on cross-border financial transactions of various countries. The financial opening result index refers to the proportion of a country’s external assets and liabilities to GDP.

For the statistics of the explained variables (real exchange rate volatilities), the real effective exchange rate index every month was calculated, which was the standard deviation of the real effective exchange rate index for 12 months in a year, and then the average value with 5 years as a node was calculated. The selection of price level is the key factor affecting the calculation of real exchange rate. Through summary, it is found that the commonly used price indexes include GDP, CPI (Consumer Price Index), WPI (Wholesale Price Index), and PPI (Production Price Index). Among them, because the consumer index is closely related to people’s consumption and life, and it is convenient to obtain the monthly data of consumer index, the real effective exchange rate index calculated by CPI was used in this paper.

The selection of control variables is mainly to control other factors that may affect the volatility of real exchange rate, such as exchange rate system, inflation rate, per capita GDP, etc. At present, the exchange rate system of each country can be divided into fixed exchange rate system, intermediate exchange rate system, and floating exchange rate system. Among them, the fixed exchange rate system has the lowest volatility, which is to keep the exchange rate fixed, and the floating exchange rate system has the biggest volatility, which is to ensure that the free volatility of exchange rate. In countries with a high inflation rate, because the domestic value of their currencies declines relatively fast, their currencies will also depreciate relative to foreign currencies, resulting in the volatility of real exchange rate increased. In this paper, the monthly CPI was used to calculate the annual inflation rate of each country. GDP per capita represents the economic development of a country, which will affect the volatility of the real exchange rate to a certain extent. Generally, for countries with more developed economies, their real exchange rate ratio is relatively stable and the volatility range is small. In addition, the devaluation of currency and the difference of productivity will also affect the volatility of real exchange rate. The descriptive statistics of the basic variables selected in this paper are shown in Table 1.

**Table 1:** Descriptive statistics of basic variables.

Variable	All country			Emerging market country			Developed country		
	Mean	Min	Max	Mean	Min	Max	Mean	Min	Max
Real exchange rate volatility	0.82	-0.64	4.01	1.29	0.29	4.01	0.42	-0.64	1.61
Total imports and exports	3.99	2.52	5.28	3.83	2.52	5.28	4.14	2.82	5.28
Trade opening policy	0.83	0	1	0.66	0	1	0.98	0	1
Financial opening policy	0.70	-1.90	2.37	-0.32	-1.90	2.37	1.60	-1.90	2.37
External liabilities	4.42	1.37	7.61	3.98	1.37	4.87	4.81	2.96	7.61
Inflation rate	4.73	4.60	6.83	4.82	4.60	6.83	4.56	4.60	5
Fixed foreign exchange system	0.25	0	1	0.11	0	1	0.38	0	1
Intermediate exchange rate system	0.60	0	1	0.75	0	1	0.47	0	1
Per capita GDP	8.95	5.22	11.46	7.71	5.22	9.66	10.03	7.68	11.46
Productivity shock	-3.72	-6.50	-1.52	-4	-6.50	-1.60	-3.48	-5.85	-1.52
Currency devaluation	0.04	0	0.40	0.06	0	-.40	0.01	0	0.20

Source: World Bank World Development Indicators (WDI) database.

### 3.2 The basic regression analysis of the impact of trade and financial opening on the volatility of real exchange rate

The correlation between the impact of trade and financial expansion on the volatility of real exchange rate was analyzed, and the relationship among the three was explored. On this basis, the pooled least squares method (OLS) was used to obtain the basic regression results.

According to the calculation results, the scatter diagram and fitting curve of the relationship between the trade opening and financial opening of sample countries and the real exchange rate volatility are drawn, as shown in Figs 3 and 4. The proportion of total import and export to GDP indicates the degree of trade opening, and the standard deviation of real exchange rate changes in 12 months of a year indicates the exchange rate volatility. It can be seen from that there is a negative correlation among trade opening, financial opening, and real exchange rate volatilities. This shows that the volatility of real exchange rate of the countries that are more in line with the integration of the world market is relatively low, and with the expansion of financial opening, the volatility of real exchange rate also decreases.

**Fig 3:** Trade opening and real exchange rate volatility.

**Fig 4:** Financial opening and real exchange rate volatility.

The pooled OLS was used to estimate the impact of trade and financial opening of sample countries on the volatility of real exchange rate in this paper. The regression results are shown in Table 2. The empirical results show that there is a negative correlation between trade opening and volatility of real exchange rate evaluated by policy indicators, while the relationship between financial opening and volatility of real exchange rate evaluated by policy indicators is not significant. From the perspective of control variables, both the fixed exchange rate system and the intermediate exchange rate system are negatively significant when the policy index is taken as the opening index. Countries with fixed exchange rate system and intermediate exchange rate system have smaller volatility range of real exchange rate than those with relative floating exchange rate system. Inflation rate, productivity difference, currency crisis and real exchange rate volatilities show a positive significant relationship. It shows that the volatility of real exchange rate is more obvious in countries with higher inflation. The change of productivity difference in China and foreign countries will affect the volatility of real exchange rate, and the depreciation of currency will also increase the volatility of real exchange rate. There is a negative and significant relationship between GDP per capita and volatility of real exchange rate, indicating that the more developed countries are, the lower the volatility of real exchange rate is.

**Table 2:** OLS regression results.

Variable	(1) OLS	(2) OLS	(3) OLS
Total imports and exports	-	-0.135	-0.198
	-	(0.0782)	(0.0791)
Trade opening policy	-0.389	-	-
	(0.0991)	-	-
Financial opening policy	0.0255	-	-
	(0.0285)	-	-
External liabilities	-	-0.0196	-
	-	(0.0560)	-
Inflation rate	0.430	0.444	0.428
	(0.131)	(0.130)	(0.129)
Fixed foreign exchange system	-0.777	-0.658	-0.670
	(0.106)	(0.117)	(0.117)
Intermediate exchange rate system	-0.175	-0.104	-0.0879
	(0.100)	(0.106)	(0.106)
Per capita GDP	-0.157	-0.164	-0.190
	(0.0318)	(0.0305)	(0.0334)
Productivity shock	0.0685	0.0733	0.0812
	(0.0387)	(0.0395)	(0.0394)
Currency devaluation	1.351	1.526	1.509
	(0.424)	(0.423)	(0.423)

### 3.3 Instrumental variable regression

Due to the endogenous problem among trade opening, financial opening, and real exchange rate volatility, the instrumental variable method was further used to estimate and get more reliable estimation results. The instrumental variables are highly correlated with endogenous explanatory variables, but not with disturbance items. Trade opening and real exchange rate volatilities affect each other. Financial opening will affect real exchange rate volatilities, and real exchange rate volatilities will affect capital flows to a certain extent. The instrumental variables of trade opening and financial opening were constructed, and the regression analysis results of sample data were obtained, shown in Table 3. The instrumental variable method is usually estimated by two-stage LS (referred to as 2SLS). First, the fitting value of explanatory variable was obtained by regression analysis, and the fitting value was regressed to the explanatory variable. The result is the regression result of LS method.

**Table 3:** Regression results of instrumental variable method.

Variable	(1) 2SLS	(2) 2SLS	(3) 2SLS	(4) GMM	(5) GMM	(6) LIML	(7) LIML
Total imports and exports	-	-1.898***	-2.339***	-2.110***	-2.614***	-2.002***	-2.602***
	-	(0.697)	(0.814)	(0.686)	(0.791)	(0.718)	(0.763)
Trade opening policy	-0.799***	-	-	-	-	-	-
	(0.372)	-	-	-	-	-	-
Financial opening policy	0.351***	-	-	-	-	-	-
	(0.128)	-	-	-	-	-	-
External liabilities	-	1.086*	-	1.285**	-	1.409**	-
	-	(0.567)	-	(0.528)	-	(0.573)	-
Inflation rate	0.779***	0.337	0.322	0.279	0.266	0.312	0.286
	(0.343)	(0.234)	(0.253)	(0.230)	(0.248)	(0.224)	(0.232)
Fixed foreign exchange system	-0.302	-0.590	-0.494	-0.675*	-0.571	-0.748*	-0.606*
	(0.196)	(0.379)	(0.354)	(0.371)	(0.348)	(0.388)	(0.355)
Intermediate exchange rate system	0.284*	0.364	0.420	0.407*	0.486*	0.419*	0.487*
	(0.171)	(0.252)	(0.281)	(0.247)	(0.274)	(0.243)	(0.262)
Per capita GDP	-0.222**	-0.249	-0.303	-0.331	-0.430	-0.418	-0.459
	(0.0903)	(0.363)	(0.408)	(0.345)	(0.383)	(0.403)	(0.422)
Productivity shock	0.0116	0.0430	0.0316	0.0393	0.0252	0.0497	0.0339
	(0.0401)	(0.0511)	(0.0532)	(0.0510)	(0.0530)	(0.0595)	(0.0603)
Currency devaluation	1.471***	0.833	0.926	0.614	0.674	0.453	0.633
	(0.533)	(0.938)	(0.962)	(0.908)	(0.933)	(0.946)	(0.909)

From the regression results in Table 3, it is found that there is a negative correlation between trade opening and volatility of real exchange rate evaluated by policy indicators and real indicators, while there is a positive correlation between financial opening and volatility of real exchange rate evaluated by policy indicators and real indicators. The inflation rate, currency devaluation, and GDP per capita are significantly positive in the financial opening evaluated by policy indicators. It indicates that the higher the inflation rate is, the more serious the currency devaluation is, the lower the GDP per capita is, and the more obvious the real exchange rate volatilities are. The countries adopting the intermediate exchange rate system are usually more likely to have significant real exchange rate volatilities than those adopting the floating exchange rate system, which is related to the fact that countries adopting the intermediate exchange rate system are more vulnerable to the impact of external exchange rate shocks, so they will face greater real exchange rate volatilities.

## 4. Discussion

Under the condition of marketization of exchange rate, the large-scale flow of international capital will impact the exchange rate, which will aggravate the volatility of exchange rate. The volatility of exchange rate will affect the financial stability from three aspects of trade, capital flow, and asset price [19]. With the improvement of financial opening, the structure of exchange rate system has changed greatly, from fixed exchange rate system to floating exchange rate system. However, for countries with imperfect financial system and insufficient foreign exchange reserves, floating exchange rate system is very vulnerable to financial risks brought by international fluid capital, especially for developing countries [20,21]. Due to the continuous implementation of China’s opening-up policy, China has been integrated into the international economic and financial market. At the same time, changes in the external market will affect the RMB exchange rate, leading to exchange rate volatilities, which will affect the financial stability and development of China. Based on this, an in-depth study and empirical test are made on the impact of trade opening and financial opening on the volatility of real exchange rate. In the era of IoT finance, data and scenarios will become new keywords. It is more forward-looking and proactive to replace collateral/pledged goods with transaction data as the first gateway to financing risk control. As a new core productivity or an innovative business model, the IoT technology will open the second curve of trade financing. In the face of noisy, dynamic, complex and high-dimensional data structures in financial markets, DL uses layer-by-layer features for feature learning: through simple and nonlinear modules to obtain features, these modules convert lower level features into a higher level, more subtle and more abstract features; then learn very complex functions by combining enough of these transformations.

With the deepening of economic globalization and world economic integration, the process and strength of financial opening up in various countries are also increasing. In the process of financial opening, it will inevitably be impacted by foreign capital, which is both an opportunity and a challenge for the financial development of China. Through the research, it is found that for all countries in the world, financial opening will aggravate the volatility of real exchange rate, but for developed countries, financial opening can reduce the volatility of real exchange rate. As a developing country, from the perspective of financial security, China should cautiously promote financial opening and guard against financial risks in the process of financial opening. At present, China’s financial opening in general is more benefit than risk, which is mainly related to China’s gradual and steady strategy. China should continue to adhere to the general idea of financial opening and economic reform, and carefully handle the risk prevention in the process of financial opening. Accurate prediction of finance and exchange rate is of great value for making effective investment strategies and risk management decisions. On this issue, the concept of DL can be introduced into the financial environment of the IoT. DL forms more abstract high-level features by recombining low-level features, which can more effectively discover distributed features hidden in data.

A deep study is conducted on the impact of the volatility of real exchange rate on the economy and the influencing factors of the volatility of real exchange rate. Then analysis is made on the impact of trade and financial openness on the volatility of real exchange rate through theoretical models and empirical studies from the perspective of opening up. Through constructing relevant models for empirical analysis, it is found that trade openness is negatively correlated with the real exchange rate volatility, and financial openness is positively correlated with real exchange rate volatility. The study of Alessandria and Choi (2021) [22] illustrated how permanent and temporary changes in trade barriers affected trade balance and how to identify changes in trade barriers, which further supports the conclusions proposed here. Kong et al. (2021) [23] reckoned that there was a long-term stable cointegration relationship between opening up and the quality of economic growth. Trade openness can significantly improve the quality of short-term and long-term economic growth. When short-term fluctuations deviate from the long-term equilibrium, the quality of economic growth can be maintained stable through automatic adjustment.

With the implementation of China’s reform and opening up, China’s trade in goods and services has been rapid development. Trade opening is not only the power to promote economic growth, but also a reliable means to maintain the stability of real exchange rate volatilities. Therefore, only by continuing to practice trade opening can the economy get steady development. However, due to the change of the world economic situation in recent years, the traditional pattern of opening-up in China has been unable to adapt to the background of the gradual rise of domestic labor cost and economic factor cost. Therefore, China should actively participate in multilateral trade system and regional trade arrangement activities, adhere to stable trade opening, promote industrial transformation and upgrading, and implement high-level trade opening policies to maintain its own trade level.

## 5. Conclusion

There is a negative correlation between trade opening and volatility of real exchange rate, and a positive correlation between financial opening and volatility of real exchange rate. The volatility in the real exchange rate can be reduced due to trade opening in the developing countries, while financial opening may intensify the volatility in the real exchange rate of the developing countries. Further study is not carried out on the logarithmic linearization and impulse response analysis, which will be further improved in subsequent studies, and the unified modeling of trade openness and financial openness will be the focus of the next stage of research.

## Supporting information

S1 Data (XLS)
